# Surgical Parapharyngeal Space Tumor Analysis with Case Series Study

**DOI:** 10.1155/2022/7083240

**Published:** 2022-02-14

**Authors:** Hani Marzouki, Mohammed Nujoom, Samiha Nezar Fagih, Razan Mohammad Almokri, Faisal Zawawi, Reda Jamjoom, Hatim Z. Almarzouki, Mazin Merdad

**Affiliations:** ^1^Department of Otolaryngology, King Abdulaziz University Hospital, Jeddah 21589, Saudi Arabia; ^2^Faculty of Medicine, King Abdulaziz University Hospital, Jeddah 21589, Saudi Arabia; ^3^Department of Vascular Surgery, King Abdulaziz University Hospital, Jeddah 21589, Saudi Arabia; ^4^Department of Radiology, Faculty of Medicine, King Abdulaziz University Hospital, Jeddah 21589, Saudi Arabia

## Abstract

**Background:**

The parapharyngeal space is a hypothetical region in the neck that stretches from the base of the skull to the bigger corner of the hyoid bone. The fascia that connects the styloid process to the tensor veli palatini separates the compartment into prestyloid and poststyloid compartments, with the prestyloid compartment being larger. In the general population, tumors of the parapharyngeal area are very uncommon, accounting for less than 1% of all head and neck neoplasms in the population. In this location, CT scanning and magnetic resonance imaging (MRI) exams are complimentary, and both tests should be performed to examine any lesions found. The most critical component of treatment is the total surgical removal of all the cancerous tissue. Identifying and treating primary parapharyngeal space (PPS) tumors are among the most challenging tasks in the treatment of head and neck cancer. They are also among the most aggressive ones. The primary goal of this study is to review our current knowledge at King Abdulaziz University Hospital, Jeddah, Saudi Arabia, which serves as an academic tertiary referral center and a major teaching center. We will focus on clinical findings, tumor structure, tumor histological distribution, and surgical approaches.

**Materials and Methods:**

The processing starts with two modules. The first module starts with the input images obtained from various patients and collected as a database. The second module starts with the collection of case series of nine patients undergoing excision via multiple different approaches: transoral, transcervical, transparotid, transmandibular, or infratemporal approach. All cases were conducted at King Abdulaziz University Hospital in Jeddah, Saudi Arabia, between 2014 and 2018. All operative interventions were performed by an otolaryngology-head and neck surgeon.

**Results:**

Our study comprised nine patients, of which two underwent transparotid and seven transcervical and combined transcervical/transparotid approach. Complications faced included a hematoma in one of our cases.

**Conclusion:**

The transcervical approach appeared to be the superior surgical approach when facing a pleomorphic adenoma within the parapharyngeal space, arising from the deep lobe of the parotid gland or parapharyngeal space-occupying paraganglioma.

## 1. Introduction

Primary parapharyngeal space (PPS) tumors are one of the most challenging tumors to be treated in the head and neck. Parapharyngeal space (PPS) is a well-known anatomical region that has the form of an inverted pyramid with a base, a vertex, and three walls. PPS tumors are considered rare tumors representing just 0.5% of all head and neck tumors [1]. The PPS is well-defined fascial space encircled by the skull base and the hyoid bone in the buccopharyngeal fascia medially and the craniocaudal axis. It is surrounded by the retropharyngeal space posteromedially and the carotid sheath posterolaterally. The fascia running posteriorly through the styloid procedure to the tensor veli palatine muscle separates the PPS into pre- and poststyloid sections. Based on the deep tumor's location in a virtual space, parapharyngeal space neoplasms (PSNs) can have a comparatively long evolution before showing some symptoms, so these tumors are likely to accomplish substantial volumes by the diagnosis time. Few arguments regarding the clinical classifications have been presented in the literature. Rifat et al. presented the lobe parotid gland tumors based on the PSNs. Hence, all of the neoplasms are not related to the deep lobe based on the PPS parotid gland. The authors suggested that few of the lesions affecting the retromandibular portion of the deep lobe based on the parotid gland must be supposed to be PSNs.

PSNs are typically indicated with medial movement based on the lateral oropharyngeal tonsil or the wall, dysphagia, cranial nerve participation, a mandibular angle mass, and pain. The PSNs are found with a stated malignant tumor rate in the range of 15–27%.

Tumors can arise mainly in the PPS, occupy it by contiguity (e.g., nasopharynx, parotid gland tumors, infratemporal fossa, and oropharynx), or arise as reserved metastases (e.g., thyroid gland, other neck and head sites, or kidney cancer). Basically, indications due to PPS metastasizing can be the first manifestation of positive primaries. Initially, PSNs are neurogenic (35–41%) or salivary (35–45%), while other histological sorts like meningiomas, hemangiomas, or lipomas are tremendously found rare. Treatment classically needs a surgical method for the PPS. Surgical approaches to PSNs are stimulating the complex anatomy, provided by the deep location and the constructions lying in the domain.

The majority of PPS tumors, approximately 80%, are of benign origin, whereas malignant tumors represent only about 20% [2]. The complexity and diverse range of analysis with various surgical methods and rarity of presentation make it intriguing to study and report these tumors [2]. The motive of this case series study is to analyze our experience at a tertiary hospital and a major teaching center at King Abdulaziz University Hospital, Jeddah, Saudi Arabia, focusing on clinical findings, morphologic type of tumors, their histological distribution, and surgical approaches.

## 2. Objective

Our primary objective in this case series is to discuss the differential diagnosis of PPS tumors at our clinical and teaching center of King Abdulaziz University Hospital, Jeddah, Saudi Arabia; to discuss the multiple approaches to a PPS tumor and the most efficient surgical methods with the least complications and the most faced complications of each approach; to compare the gender predominance in parapharyngeal space tumors; and to analyze the most commonly faced histopathology.

Literature was reviewed, and observation of our clinical and teaching center by the otolaryngology and head and neck surgeons was used later on for comparing the results with the literature to identify the best approach with the best outcomes and, all in all, the best patient survival and prognosis rates.

## 3. Materials and Methods

The current research was done on patients who presented to and were treated at King Abdulaziz University Hospital, a major multispecialty clinic and teaching hospital in Jeddah, Saudi Arabia, between 2014 and 2018, specifically focusing on malignancies that arise from structures that are situated in this anatomical region. There were a total of nine participants in the research. Following radiographic and cytological examination, all of the patients were determined to be candidates for surgical resection and received complete excision of their PPS tumors. The prediction of tumors using computerized technique is divided into two steps, segmentation and classification. Segmentation is a strategy for developing tumors in the parapharyngeal space that is based on region growth.

## 4. Results

Experiments were conducted on images obtained from hospitals to test the suggested textural feature-based parapharyngeal space tumor techniques. It was necessary to build the suggested technique using MATLAB version R2020a.

The following case series explains the stages and the various sizes of the tumor at various age groups.

**Case 1 .**

A 47-year-old female nonsmoker is presented in Figure 1 with a large nontender left-sided parotid mass. No weight loss, dysphagia, or family history of the same complaint or of any other malignancies was reported.

On examination, the mass measuring 10.0 × 8.0 cm and protruding into the oral cavity by 4.0 × 5.0 cm was palpated. It extended from the front of the auricle onto the ipsilateral side of the submandibular region accompanied by oral displacement. Neck CT with contrast showed a huge left neck mass. It is heterogeneous, does not look aggressive, and is centered mainly on the left parotid space with no visualization of the left parotid gland, the mass evidence of bony erosion. It extends deeply to the PPS compressing the oral pharyngeal airway. There were no enlarged lymph nodes, and other structures appear to be normal. True-cut needle biopsy of the parotid suggested pleomorphic adenoma. The case was presented to the tumor board. Decision was to go for a left total parotidectomy with or without mandibular split. During surgery, all parts of the facial nerve were dissected and preserved. Two level II lymph nodes were excised and sent to histopathology. Mass was excised completely using the transcervical approach, and there was no need for the mandibular split.

Figure 2 illustrates Case 1 CT images with the different cross sectional views.

Figure 3 indicates the surgical area, and Figure 4 shows the operated area. Histopathology of the mass revealed a pleomorphic adenoma and a tumor size of 11.0 × 9.5 × 5.0 cm; the lymph nodes dissected showed reactivity and were negative for malignancy.

Figure 5 shows the mass formed. The patient was discharged in good condition, tolerating oral diet well.

**Case 2 .**

A female, being 34 years of age, from Saudi Arabia, and medically free, presented to our clinic complaining of a distressing swelling in the left parotid for 1-year duration. Mass is associated with frequent discharge. In addition, there is a history of hearing impairment on the ipsilateral side. The patient denies any pressure symptoms such as dyspnea, dysphagia, and change in voice, with negative family history of the same complaint.

Upon examination, mass, measuring around 4.0 cm, with firm, immobile, and irregular edges, was visible. Palpable lymph nodes were noted on both the right and left side of the neck at level II.

Figure 6 shows the CT of the neck. It reveals a well-defined, nondestructive large mass that was noted in the deep lobe of the left parotid gland causing a pushing effect on the left external jugular vein and facial vein laterally. Furthermore, multiple bilateral enlarged cervical lymph nodes were noted at level II, with normal-appearing right parotid gland.

The case was presented to the tumor board, and consensus was to go for surgery. The patient was planned for total parotidectomy. Intraoperatively, the decision was to go with partial parotidectomy as preserving the superficial lobe was possible.

Figure 7 shows the tumor part. Through left-sided modified Blair incision, facial nerve was dissected and preserved with anterograde and retrograde techniques; the superficial parotid lobe was preserved. The mass was found to be originating from the deep lobe to the parapharyngeal space; the mass was excised. Postoperatively, there was no facial nerve weakness.

Pathology report showed a soft tissue mass measuring 5.5 × 4.5 × 3.0 cm, with an encapsulated neoplastic growth and no evidence of malignancy suggesting a diagnosis of pleomorphic adenoma.

Figure 8 shows the operated region. The patient was released in a good health condition and was followed up later in the clinic regularly.

**Case 3 .**

A female nonsmoker aged 31 years presented with an anterior neck mass with an associated lateral neck mass extending to the oral cavity for a 2-month duration, with no prior family history, no complaint of dysphagia, no change of voice, and no other neurological symptoms.

On examination, a left buccal mass and a soft palate bulge were identified with a diffuse thyroid enlargement.

Neck CT revealed a focal area of soft tissue mass noted in the left PPS, causing mass effect of the nasopharynx and on the left side fossa of Rosenmüller in the prestyloid compartment, accompanied by enlarged focal lesions in the right thyroid lobe and in the isthmus.

Figure 9 indicates all-side-view CT images. Patient's differential diagnosis included left-sided salivary gland neoplasm extending to the PPS with an associated right thyroid nodule that came back as a follicular nodule by FNA.

After presenting the case to the tumor board members, a decision was taken to perform a left-sided parapharyngeal mass excision followed by a right-sided hemithyroidectomy.

Left half apron incision was done, the PPS was approached transcervically, and the submandibular gland was excised. The lingual and hypoglossal nerves were identified and preserved. Parapharyngeal mass was identified and resected. Enlarged left jugulodigastric lymph node was observed and excised. Furthermore, a right hemithyroidectomy was performed.

Figure 10 presents the histopathology report of left parapharyngeal mass revealing pleomorphic adenoma as the clinical diagnosis. No pathological diagnosis of the submandibular gland, reactive lymphoid hyperplasia of the jugulodigastric lymph nodes, or right thyroid lobe pathological analysis was reported as follicular neoplasm.

The patient was discharged in good condition, with no complications. With ongoing regular follow-up with the head and neck team, no new events were reported.

**Case 4 .**

A 46-year-old male presented to the clinic with a left-sided neck mass for 1-year duration. No change in mass size has been observed throughout the year. The patient suffered from ongoing abundant shortness of breath and change in his vocal sound 6 months ago, with no dysphagia, no facial asymmetry, and no prior family history of the same complaint or any other malignancies. The patient has no previous history of smoking.

Neck examination showed a large, left-sided neck mass measuring 3.0 × 4.0 cm at level II; the mass was firm, mobile, not attached to the underlying skin, and nontender, with enlarged lymph nodes. Flexible laryngoscopy showed bilateral mobile vocal folds, with patent airway and normal supraglottis.

Neck CT with contrast revealed a mass encasing the inner and outer carotid arteries at the level of the separation measuring around 4.0 × 6.0 cm, eliciting lyre's sign with no airway compromise or mass effect. Features suggest carotid body tumor of the left side of the neck.

Figure 11 shows the CT scan of the head and neck. After presenting the case to tumor board members, decision was to adopt a transcervical approach; carotid body tumor was excised completely with preservation of CN XI-XII.

Histopathology report of the carotid space tumor specimen revealed a firm mass measuring 4.0 × 3.0 × 2.0 cm, all of which goes with the diagnosis of carotid body tumor, with some reactive lymph nodes.

The patient's recovery was unexciting, and he was released in a good condition.

**Case 5 .**

A male of 22 years of age presented with right-sided neck mass increasingly rising for 5 years then, becoming inferior 1 month prior to his presentation. There was no history of dysphagia, no history of facial asymmetry, and no prior family history of the same complaint or of any other malignancies.

On examination, there was a right-sided neck mass measuring 8.0 × 5.0 cm, crossing levels II & III. The mass was firm and nontender and seemed to be attached to its underlying structures. No palpable lymph nodes were felt. Fiber-optic inspection presented bilateral mobile vocal folds with no airway compromise and no intraoral bulging or mass effect.

Neck CT with IV contrast was performed, revealing an enhancing homogeneous lesion seen to extend from level of the base of skull surrounding the lateral pterygoid muscle down to the pharyngeal space. It measures 10.0 × 4.8 × 3.5 cm of height, AP, and transverse diameters, respectively.

Figure 12 demonstrates the CT scan of the head and neck in transverse structure. NA was obtained, and histopathology report showed two specimens of which one was right superficial parotid and the other was a right parapharyngeal mass. Furthermore, the patient was diagnosed with parotid tumor and another PPS lipoma. A case was discussed with the tumor board, and the decision was to go for an elective superficial parotidectomy along with excision of PPS lipoma. Through a transcervical approach and using an extended modified Blair incision, starting with the superficial parotidectomy, facial nerve identified, and retrograde dissection, all branches of it were preserved and stimulated. Then, proceeding to the lipoma of the PPS, it was identified, dissected, and excised with no major complications. Histopathological examination of the left PPS mass revealed multiple fragments of adipose tissue measuring 12.0 × 9.3 cm and resembling the lipoma with no evidence of atypia or malignancy. Right superficial parotid analysis was done; it measured 6.0 × 4.5 × 1.5 cm, with features of pleomorphic adenoma. The patient was discharged later on from the hospital in good condition, with regular follow-ups in the clinic, and showed no major new events.

**Case 6 .**

A 59-year-old man presented with a left-sided neck tumor and a tracheostomy tube, which had been put as a result of his increased shortness of breath during the previous year. The patient reported a progressive neck lump that had been growing for 17 years and had become worse in the previous two months. He became aware of a change in his voice a year ago, but his ability to swallow remained unaffected. There was a firm and nontender mass in the left side of the neck that crossed levels II-V. There were no palpable lymph nodes on the left side of the neck.

During a CT scan of the neck, it was discovered that there was a big enhancing mass on the left side of the neck, enclosing the distal half of the left common carotid artery and encasing the left inner and outer carotid arteries. As a result of pushing the oropharynx medially and generating a constriction of the airway, the carotid artery on the contralateral right side of the body was reached, superiorly spreading all the way to the base of the cranium, being 9.1 × 9.0 × 6.8 cm in length, width, and height. There were no noticeably enlarged cervical lymph nodes. The lyre's sign was clearly visible on the CT scan.

Figure 13 indicates the CT scan of the inner and outer carotid arteries by the tumor. Paragangliomas were discovered when a minor incisional biopsy was performed. The operation was completed successfully, and the patient exhibited no signs of neurological impairments while undergoing the treatment.

Our team decided to occlude the common, outer, and inner carotid arteries in order to allow for safe excision of the tumor because of its extension to the skull base and because we anticipated the potential difficulties in achieving adequate intraoperative distal control of the internal carotid artery during the procedure. Internally coiling the inner carotid artery helped to ensure that the tumor was safely removed from the skull base bone during a skull base bone excision procedure. The external carotid artery was occluded with the use of a vascular plug device in this study.

Excision of the left carotid body tumor was carried out two days after the embolization procedure was completed. The hypoglossal nerves and internal jugular vein were enclosed by the tumor. We were able to save the spinal accessory nerve, sympathetic chain, phrenic nerve, and brachial plexus throughout the procedure. During the procedure, the common carotid artery was ligated at a location near the neck, just above a coiled portion of the artery. The tumor was fully removed from the parapharyngeal region and the base of the skull. The inner carotid artery was ligated at the level of the skull base in order to prevent further damage. In addition, the tumor was separated from the contralateral carotid artery in order to completely mobilize it and enable end bloc excision of the tumor.

The patient was released in excellent health and was able to tolerate the oral diet successfully.

Figure 14 shows the carotid body tumor and internal and external carotid vessels after their complete resection.

**Case 7 .**

A 77-year-old female smoker presented with a progressive growing neck mass, complaining of a choking sensation gradually worsening over the past 3 months and associated with progressive shortness of breath and hoarseness of the voice. There was no dysphagia and no facial asymmetry, with negative family history of the same complaint or of any other malignancies.

Examination of oral cavity showed a bulge coming from the left side, with no ulceration or fungating. Palpation of the neck revealed a mobile nontender mass that is firm and solitary, measuring around 4.0 × 3.0 cm and not attached to the underlying structures or to the skin. No palpable lymph nodes were felt. Fiber-optic examination revealed bilateral mobile vocal folds with no airway compromise.

Neck CT with contrast showed a well-defined, nondestructive large mass that was recognized in the superficial and deep lobe of the left parotid gland, measuring 3.1 × 4.2 cm and causing a pushing effect on the left external jugular vein and facial vein laterally. Moreover, multiple nonsignificant bilateral enlarged cervical lymph nodes were noted. The case was discussed with the tumor board, and the decision was to go for a complete surgical excision.

The patient was prepared for total excision of the left-sided PPS paraganglioma. Through a modified Blair incision, the mass was dissected all around to the deep lobe of the parotid gland. All branches of facial nerve were preserved. Level II lymph nodes on the ipsilateral neck side were identified and dissected. Pathology report of the left parapharyngeal neck mass showed that it was measuring 2.8 × 2.5 × 1.9 cm with an irregular outer surface. The patient was discharged 2 days after the operation, and her regular follow-ups appeared uneventful.

**Case 8 .**

A 50-year-old male, previously medically free, complains of a painless localized progressive enlargement in the right side of the neck for one year. The patient does not complain of shortness of breath, stridor, cough, or dysphagia. He is nonsmoker with no prior family history of the same complaint or of any other malignancies.

On examination, there is a right-sided neck mass that measures approximately 3.0 × 4.0 cm, being rounded with a smooth surface that appears to be attached to the underlying structure and nontender mass. No visible lymph nodes were detected in the neck.

CT angiography of the neck revealed a well circumscribed mass encasing the carotid arteries at the level of the separation resembling lyre's sign. The mass measured around 4.0 × 5.0 cm, with no clear intracranial extension and no aggressive features, all of which goes with the radiological diagnosis of carotid body tumor. The case was presented to the tumor board, and the plan was to go for excision of the right carotid body tumor.

Carotid body tumor was approached transcervically, complete excision of the tumor was done around the carotid arteries along their internal and external branches. Unfortunately, internal carotid had to be sacrificed as the mass appeared to be adherent to it; however, the external carotid was preserved alongside cranial nerves XI and XII, both of which were identified and preserved. The mass was delivered completely, and a specimen was sent for histopathology. Postoperatively, the patient received one unit of PRBC due to blood loss due to the injured internal carotid artery. On histopathological examination, the mass was a firm rounded nodule measuring 4.0 × 3.0 × 1.3 cm that appeared to resemble a clear paraganglioma. The patient was discharged home after a period of observation in the hospital, and his regular follow-ups in the clinic were uneventful.

**Case 9 .**

A male of 33 years of age presented to our clinic complaining of right-sided increasing neck mass crossing the midline. The patient complaint has been ongoing for a while as he has previously been diagnosed with a right carotid body tumor case outside of our center; he had undergone a previous uncomplicated resection in 2012.

Over the last 2 months, the patient started to feel a recurring progressive right neck mass. There was no history of pressure symptoms such as dyspnea, dysphagia, or change in voice and no history of cranial nerve involvement. Review of CNS appeared to be negative. CBT prior treatment did not include radiotherapy or chemotherapy. A follow-up MRI was ordered and performed in 2013, which documented no evidence of a residual or recurrent tumor and no obvious enlarged lymph nodes with a clear operative bed.

Examination showed a 2.0 cm mass attached to the underlying muscles, being firm, immobile, and irregularly shaped. Carotid pulsations of good volume were bilaterally palpable. There was no tracheal deviation or palpable lymph nodes.

Reviewing the old histopathology report showed that a malignant glom angiosarcoma was the diagnosis in the first surgery.

An MRI of the neck was performed and revealed a right retropharyngeal carotid body space mass, lying on the same carotid bifurcation level as the previous surgery, with no invasion of the airway, and pathological right lymph nodes enlargement was observed at level III. The case was presented to the tumor board, and the decision was to undergo revision carotid body tumor excision after the embolization of the CBT with the help of the interventional radiology department. Successful embolization of the inner and outer carotid artery along with resection of the tumor was successfully done. The patient underwent CBT tumor excision through the previous cervical incision, the tumor was removed without any complication, and the carotid arteries were preserved.  Table 1 shows the preoperative examination and surgical approaches.  Table 2 presents the surgical approach and complications of the 9 patients.

The patient was discharged a week postoperatively with no complications and followed up regularly.

## 5. Discussion

PPS is a well-defined anatomical region that has the form of an inverted triangular pyramid with a base, a vertex, and three walls [3–5]. It is cut up into two sections by the tensor-vascular styloid fascia [6]. The first compartment is the prestyloid, which includes the retromandibular portion of deep lobe of the parotid gland, internal maxillary artery, inferior alveolar nerve, lingual nerve, and auriculotemporal nerve. The second compartment is the poststyloid, which contains the carotid artery; jugular vein; cranial nerves IX, X, XI, and XII; and cervical sympathetic chain [5].

Parapharyngeal space (PPS) tumors are infrequent neoplasms [3] accounting for less than 0.5% of all neoplasms in the head and neck [2]. These neoplasms may be either benign or malignant tumors with the latter accounting for only around 20% of the cases. The PPS tumors are categorized as salivary gland tumors, neurogenic and miscellaneous.

Salivary gland neoplasm is located in the prestyloid space originating from either deep lobe parotid or minor salivary gland. Pleomorphic adenoma accounts for 80–90% of salivary gland neoplasm cases, and 10–20% of cases are malignant mucoepidermoid cancer [7]. Neurogenic tumors originating in the poststyloid space could be schwannoma, which is the most common, followed by paraganglioma and neurofibroma [8]. Miscellaneous tumors include lymphoma, lipoma, hemangioma, teratoma, and liposarcoma accounting for 20% of PPS tumors [8]. Our sample of 9 patients included five men (56.0%) and four women (44.0%). All of them underwent surgery. 89% of the tumors were of benign nature whereas only 11% were malignant tumors, which is consistent with previous studies [9, 10].

The subtle symptoms of a PPS tumor make them very challenging to diagnose. Based on history, clinical examination, FNAC, and imaging, patients are diagnosed with PPS tumor, and their treatment plan includes surgical excision of the tumor [2]. At the time of diagnosis, the mean PPS tumor size was 14.1 cm, the average 20 cm, and the smallest 7.2 cm.

Initially, the majority of our patients were asymptomatic and presented only when the tumor could be detected. One of the most common marks was a neck mass. The largest tumor to be excised was 27.1 cm. The results of our study back the suggestion that PPS tumors cannot be diagnosed at an early stage. Imaging studies were used to guess the origin, side, and size of parapharyngeal tumors. In our patients, CT scan of the neck was performed in 8/9 patients and MRI in 2/9 patients. Lesions were identified in all our cases. CT and MRI were used to preview fat plane displacement and identify the relationship of the mass in association with the carotid artery. An angiography was performed in two of our cases: a case of carotid body tumor and an enhancing lesion at the carotid artery bifurcation; the latter underwent a balloon occlusion test as the internal carotid artery was planned to be sacrificed. Of these 9 sample cases, 5 were neoplasms in the prestyloid region and 4 in the poststyloid region. In all our cases, US guided FNAC was performed to control the nature of the mass, and cyto-histopathological comparison was suggested.

FNAC is a reliable procedure of precision with a relatively high specificity of malignant parotid gland tumors and provides valuable preoperative diagnostic information to the surgeon. FNAC reached 100% precision in situations where ultrasound guidance was used [11]. In order to decide on the most favorable approach, it is crucial to make an accurate diagnosis in order to safely and radically remove the entirety of the PPS tumor.

In our study, 89% of the cases were benign in origin. Of these, pleomorphic adenomas were one of the most common and accounted for 56% of the tumors. This finding is consistent with the largest systematic review performed to date, a review of 1143 PPS tumors reported over 20 years ago, which states that salivary gland tumors were the main benign PPS tumors and the most common primary lesion is the pleomorphic adenoma [12]. In our study, paraganglioma accounted for 33% (3/9), and the systemic review also had similar results as the paraganglioma was the most common neurogenic tumor accounting for 52% of the total [12].

Only one of our patients (11%) had a malignant tumor, a glom angiosarcoma. This was also consistent with the systemic review in which 18% of the tumors were malignant.

The choice of approach depends on the tumor size, the suspected malignancy, and the tumor's position with respect to the base of the skull and its relationship with the neurovascular bundle [2].

There are various surgical approaches that are suitable for resecting PPS tumors. They comprise transcervical, transparotid, transoral, and transmandibular approaches and combinations of them. (Table) Each one of these approaches has its own advantages and limitations.  Figure 15 presents a flow chart of complete preoperative examination process and surgical approaches.

The transcervical approach is the greatest commonly recognized method for poststyloid crowds appearing from the secondary salivary gland [2, 9]. Overall, the transcervical approach was most frequently performed in our cases, accounting for 67%; this is also supported by the results of the systemic review where it was the most frequent approach in tumor excision, accounting for 48% [12]. The cervical approach was used in 67% of our sample (6/9). Advantages of this approach include its superiority to the direct access of the PPS and at the carotid artery bifurcation [8, 10]; this approach has been favorable among our patients due to the aesthetic sequela [10]. On the other hand, in tumors where the superior border is near the cranial base, tumors below the inner surface of the mandible, or tumors surrounding tissue, dissection is difficult [8, 10].

The transparotid approach advocated for surgical extirpation of most deep lobe tumors [2]. This approach was only used twice in our cases: one was a pleomorphic adenoma, and the other was a paraganglioma, making up only 22% of our cases. A transparotid incision is done via a superficial parotidectomy or a face lift type incision alongside the posterior hairline for improved aesthetic outcomes [2]. This approach allows good exposure of the poststyloid compartment; this involves a total parotidectomy and extensive facial nerve dissection [13]. In this approach, a scar is usually not visible. Interestingly, when a lesion in the larger area extends to the skull base, this approach appears to be limited [10].

Transmandibular approach, also referred to as the mandibular swing/split approach, is used for high position tumors which compress the carotid artery or inner jugular vein [10]. This approach is indicated in large recurring neoplasms, large benign neoplasms, and highly vascular neoplasms where better vascular control is required [8, 14, 15]. The medial mandibulotomy transpharyngeal approach and the lateral mandibulotomy approach provide exposure and control to vascular tumors extending into the base of the skull or to oropharyngeal squamous cell carcinomas spreading into the parapharyngeal space [8, 13]. The transcervical approach is often combined with the mandibulotomy [2]. When the tumor has reached the mandible, a mandibulectomy is suggested; however, both transmandibular approaches, a tracheotomy and primary mandible repair, are needed [13]. Some surgeons might have reservations regarding potential injury to the facial, lingual, or hypoglossal nerve during osteotomy and anatomy of the soft tissue around the mandible including the chopping off of the lower lip and the temporal-mandibular articulation sub-dislocation; however, experienced surgeons might avoid such complications [5, 10].

It is possible to get better access to the PPS by the transcervical and transmandibular approaches, which allows for dissection of the primary facial nerve trunk and optimal vascular management. If necessary, the submandibular gland may be removed, and the stylomandibular ligament may be transected to provide a better working field vision. Myers and Carrau made use of this approach extensively [4]. The infratemporal approach, also termed craniofacial surgery, has been used in lesions usually involving the jugular foramen or the base of the skull with intracranial extension [2]. Transoral approach provides a direct route for the removal of small prestyloid compartment tumors which exist in the oropharynx as a bulge and do not spread into the poststyloid compartment. This approach, however, offers only limited tumor exposure and does not allow the great vessels to be controlled; thus, it is only reserved for small avascular benign tumors [5, 8, 13, 16–18]. Tumoral removal is done via the mouth through a mucosal incision over the bulging tumor [2]. Others studies have reported that the transoral approach had a 25% recurrence rate within 5 years [19]. Subsequently, a number of researchers also avoid using the approach because of the risk of damage to the blood vessels and the possible imperfect tumor exclusion [8, 20–22]. Currently, a renewed interest has emerged in robotic assisted transoral approaches and the use of Coblator to debilitate the tumor internally [2].

With more than 27 years of experience, Shahab [14] has newly published his analysis of 114 parapharyngeal tumors. Benign parapharyngeal tumor survival for 5 years and 10 years is 100%. The 5-year endurance was 93 percent for malignancies, but at 10 years it dropped to 57%. This study proved that it is improbable for a benign PPS tumor to cause mortality; consequently, it is crucial to meticulously evaluate the course of the surgical procedure and communicate with the patient [2].

The literature supported our results in other studies. A study in China [23] evaluated scientific topographies, analyses, clinical management, and handling of PPS tumors in 103 patients, of which 89 had benign tumors. The study concluded that surgery is the mainstay of treatment of PPS tumors, with transcervical approach being frequently used with the best prognosis, and that the success of the surgeries was because of the aid of imaging techniques like the CT and MRI. Another study reviewed 167 patients with PPS tumors over 10 years [24]. The study compared techniques, surgical approaches, preoperative imaging, and prognosis. Its outcomes showed that transcervical approach was the most favorable and was adopted in most of the patients, revealing good exposure intraoperatively and good prognosis with less morbidity postoperatively.

Furthermore, a study done retrospectively on PPS tumors [25] revealed that salivary gland tumors were more common than neurogenic tumors. Approaching PPS tumors transcervically was most frequently used and yielded the best prognostic results; mandibulotomy was only advocated in the presence of cranial extension.

Similarly a UAE study on 34 patients [19], with PPS tumors ranging between benign and malignant, concluded that the transparotid and transcervical approaches gave similar exposure and similar results; however, in malignant cases with extension to the cranial base, other approaches should be used such as transcervical-transmandibular, infratemporal fossa, and petro-occipital transsigmoid. However, a prospective study on 8 patients [26] suggests that the use of the combined cervical-parotid approach showed very good prognosis postoperatively, recommending the use of combined technique in more complicated cases.

Some surgical complications that could be faced during a PPS tumor resection are recurrence, hematoma, infection, fistula, facial nerve palsy, Frey's syndrome, and first bite syndrome. We faced a hematoma in one of our patients due to postoperative bleeding from an injured internal carotid artery. 89% of our patients had no complications, were cleared in acceptable condition, and were followed up regularly. From our patients, 89% were satisfied and in pleasing state and were followed up regularly with no complications.

## 6. Conclusion

The first choice for surgical removal of PPS tumors is the transcervical method due to its superiority in supply direct entry to the PPS and satisfactory control of neurovascular structures of the neck. Unfortunately, we had some disadvantages in this study. This was a backdated study with inadequate data collection and attrition rate, with limited number of cases which made statistical analysis insignificant and comparison of results between varying surgical techniques difficult. Surgical therapy of PPS tumors is difficult because of their deep position and close association with surrounding neurovascular systems. Radiological investigations of PPS tumors are required for the diagnosis and planning of surgical interventions. Excision of PPS tumors with the use of suitable surgical methods achieves favorable results.

## Figures and Tables

**Figure 1:** A photograph showing an oral bulge in left lateral side wall of the oropharynx.

**Figure 2:** (a, b) Axial cut CT images showing the heterogenous left-sided smooth surface mass with minimum mass effect on the oropharyngeal airway, with no destruction of the mass and no intracranial extension. Mass appears to be around 10 cm in size. (c, d) Coronal cut CT images showing the mass from the left side with no mass effect on oropharyngeal airway.

**Figure 3:** Patient in the operating room with markings for mandibular split, but intraoperative decision was to go with transcervical and transparotid combined approach.

**Figure 4:** (a) Branches of the facial nerve, being fully intact and preserved, can be seen over the mass. (b, c) Mass dissected and fully delivered. (d, e) Defect can be observed all the way into the parapharyngeal space with full preservation of facial nerve and its branches.

**Figure 5:** Mass fully dissected and delivered to histopathology.

**Figure 6:** (a–c) Axial cut CT images showing the heterogenous left-sided smooth surface mass with minimum mass effect on the oropharyngeal airway, with no destruction of the mass and no intracranial extension. Mass appears to be around 10 cm in size. (d–f) Coronal cut CT images showing the mass from the left side with no mass effect on oropharyngeal airway.

**Figure 7:** (a–d) Tumor cautiously resected while fully preserving the facial nerve. (e, f) Facial nerve fully intact over PPS defect. (g, h) Defect can be seen through the PPS.

**Figure 8:** Mass fully delivered and sent to histopathology after superficial parotidectomy.

**Figure 9:** (a) Axial cut CT images revealing left-sided PPS. (b, c) Coronal cut CT images showing the PPS arising from the deep lobe of the left parotid. (d) Minimal mass effect of the tumor on the oropharyngeal airway.

**Figure 10:** Purely transcervical approach with release of stylomandibular ligament to achieve adequate exposure.

**Figure 11:** (a, b) CT scan of the head and neck revealing mass encompassing the inner and outer carotid arteries at the level of the bifurcation.

**Figure 12:** MRI of the neck reveals an enhancing homogeneous lesion seen to extend from level of the base of skull surrounding the lateral pterygoid muscle down to the pharyngeal space down to the lower neck level of the cricoid cartilage. Mass appears to measure 10.0 × 4.8 × 3.5 cm of height, AP, and transverse diameters respectively.

**Figure 13:** (a) An axial CT image showing the complete engulfment of the inner and outer carotid arteries by the tumor. (b) A reconstructed coronal image showing the tumor's extension to the skull base. (c) An angiogram showing splaying of the inner and outer carotid vessels (lyres sign) and tumor blush. (d) A postembolization picture showing the coils in the left common carotid artery (star) and in the left internal carotid artery above the skull base (arrow), and the vascular plug in the left external carotid artery (circle).

**Figure 14:** The carotid body tumor and internal and external carotid vessels.

**Figure 15:** Schematic depicting the preoperative examination and surgical approaches of the PPS tumors.

**Table 1:** The preoperative examination and surgical approaches of the PPS tumors.

No.	Sex/age	Year of treatment	Histopathology	Site	Size (cm)	Imaging	FNAC
1	F/47	2017	Pleomorphic adenoma	Prestyloid	10.5 × 10.0 × 6.6	CT	Yes
2	F/34	2017	Pleomorphic adenoma	Prestyloid	5.5 × 4.5 × 3.0	CT	Yes
3	F/31	2017	Pleomorphic adenoma	Prestyloid	5.0 × 2.7 × 4.0	CT	Yes
4	M/46	2018	Pleomorphic adenoma	Prestyloid	4.0 × 3.0 × 2.0	CT/contrast	Yes
5	M/22	2015	Pleomorphic adenoma lipoma	Prestyloid	6.0 × 4.5 × 1.512.0 × 9.3	CT/IV-contrast MRI	Yes Yes
6	M/59	2016	Paraganglioma	Poststyloid	9.1 × 9.0 × 6.8	CT/angiography	Yes
7	F/77	2015	Paraganglioma	Poststyloid	2.8 × 2.5 × 1.9	CT	Yes
8	M/50	2018	Paraganglioma	Poststyloid	4.0 × 5.0	CT	Yes
9	M/33	2016	Glomangiosarcoma	Poststyloid	5.3 × 4.5 × 3.1	MRI	Yes

**Table 2:** Surgical approach and complications of the 9 patients.

No.	Surgical approach	Complications
1	Transcervical and transparotid	None
2	Transparotid	None
3	Transcervical	None
4	Transcervical	None
5	Transcervical	None
6	Transcervical	None
7	Transparotid	None
8	Transcervical	Bleeding
9	Transcervical	None

## Data Availability

The data that support the findings of this study are available on request from the corresponding author.
